# Analysis of the Influence of Geographical Environment on Chinese Ethnic Folk Dance, Taking the Development of Dance Curriculum in Huaihua No. 1 Middle School as an Example

This article has been retracted.

**DOI:** 10.1155/2022/9692803

**Published:** 2022-08-29

**Authors:** Xin Liu, Young Chun Ko

**Affiliations:** ^1^College of Music and Dance, HuaiHua University, Huaihua City, Hunan Province 418008, China; ^2^Daprtment of Education, Graduate School of Sehan University, Chonnam 58447, Republic of Korea; ^3^Department of Teaching Profession, Sehan University, Chonnam 58447, Republic of Korea

## Abstract

Among the treasures of Chinese art, ethnic dance is an important part. As a key form of expression of national art and emotion, dance has strong regional and gender characteristics for those affected by different ethnic groups and regions. The unique characteristics of the region are the driving force for the masses of all ethnic groups in China to continuously promote the prosperity and development of ethnic and folk dances living alone in different living conditions and living environments. In the analysis of ethnic and folk dances, environmental elements have a profound impact on the rapid development of dance. The main reason for folk dance is the relationship between the costumes of the dance, the connotation of the dance, and the laws of nature, resulting in the derivation of the environment. The article will also focus on a more in-depth discussion and analysis of the characteristics of Chinese folk dance. Scientific research on the regionality of ethnic dance plays a vital role in understanding and inheriting ethnic and folk dances.

## 1. Introduction

Folk dance is a traditional Chinese art genre that is loved by people and shows richness and diversity in the form and content of dance. In the establishment of the dance, the environmental hazard dance content is created [1]. The deepest elements give Chinese folk dance distinctive dance characteristics, which can better promote the research and development of the influence and value of Chinese folk dance [2].

Chinese folk dance is an integral part of China's outstanding traditions. The regional scientific research of folk dance is conducive to carrying forward and inheriting the excellent Chinese tradition and promoting the rapid development of the tradition in the new era [3]. In the process of inheritance and development, Chinese folk dance has constituted distinct national characteristics and local culture, with the unique charm of atmosphere, popularity, challenge, and beauty [4]. Folk dance is one of the manifestations of the locals. It is influenced by a variety of environments and living customs, and is closely related to the special regional environment [5].

At present, in the cultivation of national and folk dance talents, professional colleges and universities use the training system of classical ballet, classical dance, and modern dance blocks [6]. In terms of posture, sense of rhythm, technical skills and other aspects, the training obtained by students cannot be directly used for the teaching and performance of ethnic folk dance courses, and must be restored through the shaping of national folk dance styles. Taking the Beijing Dance Academy and the Inner Mongolia Academy of Arts as pioneers in exploring the “basic training of Chinese folk dance,” the teaching content of the “Basic Training of Ethnic Dance” of the Beijing Dance Academy belongs to the typical folk dance body shape and flexible rhythm [7]. The advantage of this innovative curriculum is that it can break through the traditional course content, create its own unique course content, and define the rhythm, method and technique of folk dance. [8] Inner Mongolia Academy of Arts serves as a training base for Mongolian dance writing and performance. [9] Based on the diligence of many generations, the Mongolian Language Skills Training Textbook was released, and the basic skills management system of Mongolian dance was established and optimized [10]. The exploration and practice of the discipline has played a positive role in enriching and optimizing the Teaching System of Chinese Folk Dance [11]. The basic skills of folk dance practice are a very inquiry-based dance basic training method, with a certain degree of innovative ability [12]. The existing experience and achievements of the Beijing Dance Academy and the Inner Mongolia Academy of Arts have brought basis and reference to the basic training of Cangyuan Wa folk dance [13].

A revitalized, prosperous, and strong country [14]. National dance is the essence of the Chinese nation and embodies the development of literary and artistic styles and spiritual outlook of all nationalities. Ethnic dance is one of the main courses of higher teacher dance studies. [15] General dance science should dig deep into the true meaning of ethnic folk dance, give full play to the advantages of folk dance, and cultivate the inheritance and development of students' professional dance skills [16]. Therefore, promoting the application and practice of ethnic folk dance in the higher teachers' dance curriculum plays a crucial role [17]. The article will also carry out more in-depth discussion and analysis of the characteristics of Chinese folk dance. The scientific study of the regionality of ethnic dance plays a vital role in understanding and inheriting ethnic folk dance.

## 2. The Development Status of Chinese Folk Dance

### 2.1. Characteristics of the Development of Folk Dances

#### 2.1.1. Environmental and Folk Dance Formation

Geomorphology, climate, natural scenery, and other factors lead to different types of natural environments. In China, Mongolia has been known for singing and dancing since ancient times. They like to express their affection for life according to national dances, so their personalities are extroverted and pure. Because of the weather, the climate was dry and the rainfall was low, and they often traveled according to the waterway, but the Inner Mongolian grasslands were open to the horizon and more open to emotions. Therefore, the vast majority of Mongolians in Wuhan are bold and rude day and night, and feel absurd pride. In addition, the Mongolian steppe life is closely related to horses, and can often be seen in Mongolian dances [18].

#### 2.1.2. Geographical Characteristics and Characteristics of Folk Dances

Each place produces a different ecology, especially in folk dances. For example, the Mongolians in Wuhan are engaged in livestock herding, hunting, production and manufacturing day and night, and have lived in the vast grasslands for a long time. Sheep refers to the life of the Mongol Huns. In addition, “fall dance” and “wooden chopsticks” are very characteristic dances of the Mongolian people. This dance posture is casual, there is no certain dance regulations, but the dancer must mainly express the rhythm, rhythm and body language of the Mongolian people in Wuhan. Mongolian people in Wuhan are enthusiastic and bold. In general, Mongolian dance is influenced by the environment, and its unrestrained, enthusiastic and unrestrained characteristics are closely related to the steppe [19].

#### 2.1.3. Geographical Characteristics and Changes of Ethnic Dances

The national customs with different characteristics are very different, which is especially evident in China's folk dances. For example, Mongolia in the northern region of Wuhan is a vast area that is day and night, prompting folk dances to be more vivid, diverse, and enthusiastic. On the other hand, because the Yi people in Wuhan in the southern region are more likely to splash around Wuhan day and night, their folk dance is soft, delicate, and beautiful. From this point of view, the natural environment has a great influence on folk dance. Different characteristics will form different types of folk dances. Along with the development of society and science and technology, folk dances were disseminated according to science and technology. In addition, the spread of folk dance is continuous and multidimensional. Therefore, in the development of folk dance, the people of all ethnic groups need to accept better and beneficial things and promote the common development of the people of all ethnic groups [20].

### 2.2. Development Trend of Folk Dance

#### 2.2.1. The Specialization of Folk Dance is Gradually Strengthened

Folk dance not only stipulates that dancers have strong theoretical knowledge, but also requires them to constantly improve themselves in the performance process. In that way, it will get strong support and love from more audiences. In addition to this, folk culture can also be described in a unique way of folk dance. Therefore, when carrying out national dance performances, dancers only need to have more professional dance skills to better present the national style and gain a wide audience. Great support and recognition from good friends [21].

#### 2.2.2. Folk Dance Should Follow the Footsteps of the Times

Under the premise of inheriting, developing and maintaining folk dances, we should be soberly aware that we must inherit, develop, and maintain folk dances to make them stronger. Only by closely integrating with the spiritual essence of national dance and pioneering and innovating can Chinese national dance develop continuously and for a long time. We should keep pace with the times and absorb the dross of folk dance under the premise of innovation, and inherit and develop folk dance stronger and more comprehensively.

#### 2.2.3. Diversified Development of Folk Dances

In our country, there are clear differences among the various ethnic groups. Because of these differences, folk dances constitute a variety of performance forms. Under the premise of retaining the advantages of folk dance, a variety of performance forms should be combined with the advantages of other dances, and the folk dance is advancing with the times. Highlight the unique charm of folk dance. Only in this way can the diversity of folk dance be realized.

China is a vast country, with a vast area from north to south, a vast area of goods, and a variety of ecological environments. Wuhan people key to live in the vast central plains area, other brothers and ethnic groups are key distributed in the nearby areas. The vast majority of China belongs to the subtropical and temperate climate, and a very small number of areas belong to the tropical monsoon climate, so the vast majority of areas are suitable for the development trend of agriculture and other crops. The distinctive environment and natural conditions have made it possible to form a traditional style in China based on the agricultural economy and the Han people, and also produce a wide variety of folk dances of various ethnic groups.

In general, the folk dances of various ethnic groups in China are key to the areas inhabited by various ethnic groups, but due to the identity of languages and customs, as well as the exchange and combination of various ethnic groups in the process of migration, it constitutes a dance between ethnic groups and regions. Dance form. This very distinctive characteristic and the current situation of individual and continuous communication and development of various ethnic groups are the distribution of Chinese national folk dances (Figure 1).

Compared with the Han Chinese, the number of other fraternal ethnic groups is significantly scarce, but the housing area of 50 yuan accounts for the total area, the straight-hair splint Dili Lonzo accounts for the total area, and the 60 yuan accounts for the total area. The key exists in the northeast region, Inner Mongolia, the great northwest, the southwest region, central China, and parts of the southeast. A long-term nomadic herder of mongolian, Uzbek, and other ethnic groups settled in the vast steppes of the north, their dances embody the life of nomads riding horses. The muscles of this dance are stiff but rhythmic. The folk dances of the Zhuang, Wa, Hani, and other ethnic groups in the agricultural and pastoral areas of the southern region mainly show the working life of picking tea and washing rice, with soft postures and a sense of rhythm. The folk dances of various nationalities living in the border areas of the motherland have socialist democracy, and there are many similarities or similarities with the dances of different nationalities in close proximity abroad. In addition, in special areas, the ancient Chinese cultural assets of folk dance are more abundant. For example, the folk dances of the Uighurs and other ethnic groups on the Silk Roads applied the technicality of the head and waist, exposing the dance property of the ancient Western Regions.

### 2.3. Principles of Application of Ethnic Folk Dance in Dance Courses

#### 2.3.1. Principles of Innovation

With the progress and development of the times, the public's artistic aesthetic ability has improved. As a traditional art method, folk dance must pay attention to the standard of artistic innovation when applied to the classroom teaching of the physical fitness class of the senior teacher. The specific content of art is constantly innovated with the development of the times, presenting the characteristics and imprints of the times, and conveying the feelings and ideas of the times. Folk dance is also in the development stage. Some national dance arts have been inherited and developed, and some national dances have undergone new changes along with the development of the times. The use of folk dance in the dance curriculum of colleges and universities must explore the uniqueness of folk dance from an innovative perspective, and closely integrate with modern dance art, only innovation can continue to carry out the heavy responsibility, and can attract teachers in the new era.

#### 2.3.2. Principles of Practicality

Dance is a highly theoretical course content that must teach students dance skills and practical body shape skills. As a kind of dance plastic art, folk dance has rich and diverse artistic value and more professional dance methods. That's an integral part of the dance line. In that case, attention should be paid to the applicability of folk dance in the higher teachers' dance classroom. On the one hand, in the folk dance repertoire, it is necessary to select representative folk dances to allow students to increase their insight and guide students to grasp dance skills. On the other hand, in the practice of national folk dance, it is necessary to have both the characteristics and methods of national folk dance, combined with other dance elements, to create a distinctive dance and enhance the viewing value of national folk dance.

#### 2.3.3. Artistic Principles

Folk dance is an important form of plastic art, and different ethnic groups have different dance forms. The use of folk dance in higher teacher training dance classes should follow expressiveness. In the process of teaching ethnic and folk dance, teachers should dig deep into the expression of ethnic art that is often contained in dance, so that students can have a deeper understanding of ethnic minorities, art and characteristics, and then firmly grasp the art and characteristics of ethnic dance. At the same time, the teacher wants the students to learn to independently discover, learn, and apply the artistic characteristics of ethnic minority dance to create new dance art forms.

## 3. Development Concept of Chinese Folk Dance Curriculum

This scientific research is committed to the flexible use of the theoretical knowledge and methods of ethnic dance, sociology, ethnology, art aesthetics, and other disciplines to grasp the cognition and behavior of children in Chinese folk dance at this stage, and to explore and analyze the multiple elements that affect their formation. The author's research process begins with extraordinary reflections. From shallow to deep, integrating social experience and theoretical analysis, I give a variety of assumptions that harm children's cognitive ability, performance and evaluation of Chinese folk dance. Subsequently, if this is transformed into a series of measurable problems. Using sociological and psychological research methods, the questionnaire is carried out according to the design principle of the questionnaire method, and reasonable special tools can be selected to complete distribution, recycling, analysis, and collation. Ultimately, investigation and scientific research can coexist. According to a reasonable level, the research subjects were selected and the survey samples were obtained from the designated addresses. Therefore, this chapter focuses on the three key steps that the authors customize in the subject research: research hypothesis, research methods, and research objects.

### 3.1. Research Subjects

In the end, the author chose Huaihua No. 1 Middle School as the research address. Huaihua No. 1 Middle School was established in 1943. In 1979, it was identified as the first key middle school in Huaihua City, and in 2002, it was selected as a key middle school in Hunan Province. In 2007, the high school and middle school were separated, and it became an independent high school. At present, it covers a total area of 42,300 square meters with a total construction area of 24,400 square meters on campus and a total area of 63,300 square meters for a large school farm. At this stage, there are 39 classroom teaching groups, 1922 students, 197 active teaching staff, 181 full-time teachers, 169 teaching teachers (accounting for 85.78% of the teaching staff), including 13 graduate students (accounting for 7.69% of the teaching staff), 1 specialist teacher, 1 senior teacher, 66 senior teachers, and 96 first-level teachers. The teaching content of the ethnic folk dance course of Huaihua No. 1 Middle School is shown in Figure 2.

From September to November 2017, the author conducted a sample survey of students at Huaihua No. 1 Middle School. A total of 526 questionnaires were searched, of which 518 were valid, and the effective rate of questionnaires was 98%. The sample reflected the different characteristics of respondents in five areas: gender, race, place of origin, occupation type, and household income. The basic information is shown in the following table (Table 1).

### 3.2. Frequency Domain Analysis of the Survey Results

The above research design introduces the “Survey on the Recognition of Chinese Folk Dance by Primary and Secondary School Students”. 30 puzzles, recycling effective questionnaire 518 copies. Brief analysis, narrative, and data analysis of four-dimensional databases are the focus of this chapter. Xiaobian mainly expounded the frequency domain of each recognized dimension database from a macro perspective, selected a representative topic to discuss, and proposed a survey report in the form of data charts. According to the results of the four basic dimensions, the overall observation of the cognition of Chinese folk dance by college students, the shortcomings of the frequency domain are found, and the clues for detailed analysis and reflection are reported.

#### 3.2.1. Emotional Preferences

Selected by college students in the research on the emotional level of Chinese ethnic folk dance. “What kind of folk dance do you like?” What are the key reasons? At the level of content and style, I came to investigate children's interest in learning Chinese folk dance. The results of these two multiple choice questions can be clearly seen from the pie chart below (Figure 3).

According to the statistical analysis of time-domain data in the survey report above, the overall conclusion of emotion in terms of identifying with the four dimensions of Chinese folk dance exceeded expectations. Specifically, it is manifested in the high preference for Chinese folk dance, the overall impression preference, different ways, specific content, and design style of the need for diversification of dance works.

#### 3.2.2. Cognitive Definitions

In the questionnaire survey, there is a problem in the cognitive dimension of Chinese folk dance among college students. Can you clearly distinguish between Chinese folk dance and other dance styles? In other words, investigate whether college students can clearly identify dance styles. In order to distinguish whether the difference between Chinese folk dance and other dances can be accurately distinguished, the creator first hoarded his own cognitive discrimination. The details are as follows (Table 2).

According to the frequency domain analysis of the two problems of cognitive dimension, it is not difficult to find that most college students have a poor and unclear understanding of the dance types and ethnic definitions of Chinese folk dance, and a considerable number of students have a lower cognitive level than them. In addition, it is possible to look for clues to the case of the behavioral dimension. Finding the final two problems, college students' awareness of professional classics is not too high, and the contact area is narrow.

#### 3.2.3. Evaluation Status

This article explores the most intuitive evaluation of Chinese folk dance by college students. The author mainly uses five levels of satisfaction to measure viewing experience and development satisfaction. The distribution of data for these two aspects is shown in the following table (Table 3).

From the above table, we can observe the evaluation and development attitude of college students on national folk dance works. What can be improved in these two areas? College students also gave their opinions through two questions: “What kind of folk dance works do you want to see in the future?” And “In what way do you think Chinese folk dance should be passed on?” “Comments, because both questions are multiple choice, the following two bar charts (Figures 4 and 5) show the results of this survey.

Based on the above data, the recognition of Chinese folk dance by college students in the evaluation dimension is as follows: First, the overall viewing evaluation is good, and the satisfaction with the current national folk dance works is relatively high; Second, public participation in square folk dances, higher dance types have higher attention and uneven evaluations. However, they are not satisfied with the current development status of national folk dance, and have their own thoughts and worries about the future development direction of national folk dance.

## 4. Summary of Survey Results and Countermeasure Studies

### 4.1. Summary of Survey Results

Based on the time domain, classification, and difference analysis of the survey report, we basically understand the current status and factors of the students' identity at this stage. After considering and understanding the correlation between dimensions, the survey report can be summarized below

1. Under the recognition of the four dimensions of Chinese folk dance, college students showed their preference for the emotional dimension, insufficient thinking ability, weak relativeness of personal behavior, and different evaluation standards.
2. All in all, college students' preferences for folk dance focus on the diversity of methods, specific contents, and design styles, and the acceptance of various types of folk dances is relatively high, and it is expected that there will be more interesting and better quality folk dances. The work takes place.
3. College students want to spread folk dances to foreign friends more than they meet foreign friends. As Felix “livin” it home it gross often says, the bridge between the “land (in a sense, morphological consciousness)” forms this precondition, the necessary dual identity. Second, this identity is identity, which is equivalent to the identity of the state. This identity is very clearly reflected in citizenship. Thus, Chinese citizenship rules and regulations constitute two or more legal and philosophical ways of defining identity. Such identities are mutually exclusive and mutually reinforcing, not conflicting.”
4. According to the investigation of college students' cognition and appreciation of Chinese folk dance works, it was found that there were significant differences in the works displayed on different service platforms. The national folk dance works performed on CCTV's “Spring Festival Gala” and other platforms are very easy to enter the eyes of the masses and audiences, and it is very easy to develop and win the hearts of the people. Although other professional dance competitions and website platforms are very low-profile, there are already many outstanding classics. Therefore, the audience of these channel columns is usually more professional and has a better understanding and recognition of folk dance.

### 4.2. Countermeasure Research

#### 4.2.1. Cultural Output to Enhance Self-Confidence

Global, imported and exported, singleness and pluralism, contention, and resonance. From the 1990s, the impact of economic globalization on human society has been expanding in all aspects. We do not know the combination of this association. We have to spread the innovation. Output rates are not only a major indicator of international status and ability to innovate, but also a way.

With a strong support platform and good feedback on the actual effect, deriving the traditional sense of belonging and confidence in Wuhan is really the most appropriate countermeasures and suggestions to integrate into the inherent requirements of the current situation and strategic development plan. It is hoped that their folk dances can rely on this fashion trend to show their brilliance to the world in more diverse ways. It is hoped that college students will have more opportunities to participate in the opening up and popularization of national dance.

#### 4.2.2. Strengthen the Gripper and Create Symbols

Cultural symbols are the unique extraction and abstract reflection of a region, a nation, and a country, carrying extremely rich and long-term connotations. Just like time to go to China first, see the United States Hollywood think of the United States, see the cherry blossoms think of Japan. Symbols are conducive to understanding different connotations, and we can easily identify the characteristics of different places according to symbols. If China's 56-piece national dance has unique symbols, can everyone understand it more clearly? For ethnic and folk dances, the better representative is the symbolic posture of various ethnic regions. In the development and popularization of Chinese folk dance, this representative movement can be established and implemented at all levels.

#### 4.2.3. Policy Guidance, Education First

All cultural education should be gradually from children, and the enlightenment education of folk dance is not as good as the content of other scientific and educational courses. Mainly because the education that plays an important role in the Chinese folk dance, the curriculum seems to be blank. Fortunately, the state has paid more and more attention to comprehensive quality education, and various literary and artistic classes have sprung up on campus. Folk dance can take this opportunity to enter the primary and secondary school curriculum. Some have already taken the lead. For example, some HLTs in Yushu, Qinghai, use Tibetan dances instead of radio exercises. Even if it is a primary school in Guangdong Province, the class is also inspired by Yao Zongzong. Hubei Enshi No. 5 Middle School Hubei Laifeng a number of primary and secondary schools to carry out traditional opera into the campus theme activities. This different teaching method constantly improves the curriculum system of Chinese folk dance.

## 5. Conclusion

In general, folk dance is developed in a different regional natural environment, and regionality is the most basic feature of folk dance. As one of the main characteristics of folk dance, regionality not only shows different types of national characteristics, but also shows a strong national charm and living customs, which is a very important material and spiritual capital for the people. The rapid development of a nation is inseparable from the far-reaching influence of the local environment. A variety of folk dances have been derived from national characteristics. The ethnic dances of various nationalities constitute their own unique dance styles, forming a brilliant and rich and diverse Chinese tradition.

## Figures and Tables

**Figure 1:** Development trend of major performance types in China in 2021.

**Figure 2:** Teaching content of ethnic folk dance course in Huaihua No.1 Middle School.

**Figure 3:** Pie chart of the type of folk dance works that college students like.

**Figure 4:** Students' expectations for folk dance works.

**Figure 5:** Expectations of college students for the development of ethnic and folk dances.

**Table 1:** Basic information of secondary school students' ethnic and folk dance identity survey subjects (*N* = 518).

Basic functionality		Number	Percentage%
Sex	Male	164	31.66
	Female	354	68.34

Nationality	Chinese	392	75.68
	Ethnic minorities (21 in total).	126	24.33

Place of birth	Cities inhabited by ethnic minorities	110	21.24
	Rural areas inhabited by ethnic minorities	30	5.79
	Cities where there are no ethnic minorities living	288	55.60
	Rural areas in non-ethnic minority areas	90	17.37

Professional	Natural science	116	22.39
	Social science	402	77.61

Household income	2300 or less	84	16.22
	2301–6000	208	40.15
	6001–10000	122	23.55
	10001–15000	40	7.72
	More than 15001	64	12.36

**Table 2:** Students' self-judgment on Chinese folk dance cognition.

Cognitive dimensions	Number	Percentage%
Very clear	62	11.97
Relatively clear	168	32.43
Unable to distinguish	158	30.5
Uncertain	112	21.62
Very unclear	18	3.47

**Table 3:** Direct evaluation of Chinese folk dance by college students.

Two aspects of different dimensions of the survey	Watch the experience (%)	Development assessment (%)
Very good	33.59	6.65
Better	46.72	30.5
Unable to distinguish	16.99	42.47
Not so good	1.93	19.31
Very poor	0.77	0.77

## Data Availability

The labeled data set used to support the findings of this study is available from the corresponding author upon request.
